# Invasive Streptococcus agalactiae Disease With Meningitis and Septic Arthritis in a Non-pregnant Patient

**DOI:** 10.7759/cureus.31077

**Published:** 2022-11-04

**Authors:** Telmo Coelho, Maria Pacheco, Tiago Mendes, João Valente, Pedro Gil

**Affiliations:** 1 Internal Medicine, Centro Hospitalar Vila Nova de Gaia/Espinho, Vila Nova de Gaia, PRT; 2 Internal Medicine, Hospital Sousa Martins - Unidade de Saúde Local da Guarda, Guarda, PRT; 3 Medicina, Hospital Conde de Bertiandos, Unidade Local de Saude Do Alto Minho (ULSAM), Ponte de Lima, PRT

**Keywords:** streptococcus agalactiae meningitis, streptococcus agalactiae, septic arthritis, meningitis, group b streptococcus agalactiae bacteremia

## Abstract

*Streptococcus agalactiae* is a common constituent of the human flora. However, infection in immunocompetent adults is uncommon and the involvement of the central nervous system (CNS) or development of septic arthritis are exceedingly rare and by our knowledge, were only described simultaneously once in a retrospective study.

We present the case of a 66-year-old woman with *S. agalactiae* bacteremia presenting meningitis and septic arthritis of the left shoulder. The patient presented to the emergency department with altered mental status and fever. Lumbar puncture revealed cerebral spine fluid (CSF) pleocytosis and elevated proteins. Blood and CSF cultures identified the presence of a susceptible strain of *S. agalactiae*.

During hospitalization, the patient complained of left shoulder pain, enabling the identification of articular fluid collections, which were drained confirming their infectious origin. Colic ulcers were found to be the starting point of this infection with posterior involvement of the CNS and the development of septic arthritis by hematogenous dissemination.

## Introduction

*Streptococcus agalactiae*, a gram-positive coccus bacterium, is a common constituent of the normal flora of a human. It is primarily found in genital flora and eventually transmitted during labour and delivery, resulting in the colonisation of the baby [1]. Therefore, *S. agalactiae* infections are more common in pregnant women and neonates [2]. In some cases, it can cause bacteraemia in non-pregnant adults, mostly in immunocompromised hosts and patients with hepatic or renal failure [3].

However, the involvement of the central nervous system (CNS) or development of septic arthritis is exceedingly rare, and to our knowledge, was only described simultaneously once in a retrospective study [4]. In fact, in large cohort studies only 0.4% to 7.4% of bacterial meningitis were caused by *S. agalactiae*, usually associated with one of three predisposing conditions: immunocompromised patients, cerebral spinal fluid (CSF) leakage or extra meningeal sanctuary, like an abscess or endocarditis [5-7].

Septic arthritis due to *S. agalactiae* remains rare, being responsible for only 5%-10% of all septic arthritis [8,9]. Large retrospective studies found that articular involvement was associated with predisposing conditions, such as immunosuppressive diseases or vaginal colonization at the time of delivery [8,9]. Knee and shoulder joints were found to be more commonly affected [8,9].

## Case presentation

We present the case of a 66-year-old woman admitted to the emergency department (ED) with altered level of consciousness in the last 24 hours characterized by confusion and disorientation. She had a past medical history of hypertension, dyslipidaemia, being overweight, and alcohol consumption of 50 grams per week.

On physical examination, she was disoriented and had disorganized speech. She also had mild abdominal tenderness, but the evaluation was otherwise unremarkable, notably Kernig and Brudzinski signs were negative. She had a fever (body temperature of 38.3 degrees Celsius), normal blood pressure (122/73mmHg), heart rate (83 beats per minute) and oxygen saturation level (98% at room air). Blood tests performed in the ED revealed leucocytosis (9,470/µL) with neutrophilia (86%), and an elevated C-reactive protein level of 17.38mg/dL. Blood urea nitrogen (BUN) and liver function tests were normal. A head computed tomography (CT) scan showed no signs of increased intracranial pressure or other abnormal results. A lumbar puncture was performed which revealed pleocytosis (14 leukocytes, 50% polymorphonuclears) and high protein levels (662/µL).

Blood cultures were collected and empirical antibiotic therapy with Ceftriaxone, Ampicillin and Acyclovir was started, with the patient being admitted to the Internal Medicine Department. A susceptible strain of *S. agalactiae* was later identified in cerebrospinal fluid as well as in blood cultures, which allowed us to de-escalate antimicrobial therapy to Ampicillin alone.

The diagnosis of *S. agalactiae* bacteraemia with meningitis was clear but we still struggled to find an explanation for this infection in an immunocompetent and non-pregnant woman without previous history of head trauma or neurosurgical interventions. To exclude diseases associated with immunocompromise, viral serologies (HIV, HBV and HCV) were performed, which were negative. A complete cervical, thoracoabdominal and pelvic CT scan found no abnormalities.

During the first week at the hospital, the patient complained of abdominal pain, diarrhoea and haematochezia. She underwent endoscopic examinations: revealing a normal upper gastrointestinal endoscopy and a colonoscopy presenting ulcers with irregular edges in the sigmoid colon, without bleeding stigmata. Biopsy of ulcers confirmed an infectious aetiology, allowing us to presumably consider the colic ulcers as the primary source of the *S. agalactiae* infection. CNS involvement was probably due to hematogenous dissemination.

At this time, the fever recurred, and the patient started to complain about left shoulder pain, swelling and movement limitation. New blood cultures were collected, and antibiotic therapy was switched to Ceftriaxone. Articular ultrasound (Figure 1) showed hypoechogenic fluid collections, which were confirmed by CT (Figure 2).

**Figure 1:** Left shoulder ultrasound revealing hypoechogenic fluid collections.

 

**Figure 2:** Left shoulder CT scan showing hypodense fluid collections.

The patient underwent ultrasound-guided arthrocentesis (Figure 3) and articular debridement. Fluid analysis (90.413/µL leukocytes, 95% polymorphonuclear) substantiated the diagnosis of septic arthritis. Nevertheless, blood and articular fluid cultures were negative.

**Figure 3:** Ultrasound-guided left shoulder fluid drainage.

After a multidisciplinary team meeting, we concluded that an invasive *S.s agalactiae* infection with primary source in colic ulcers, resulting in bacteraemia and haematogenous dissemination causing CNS and articular affection, was the most likely diagnosis. After six weeks of directed antimicrobial therapy, the patient had a complete resolution of confusion and shoulder pain and did not have any gastrointestinal complaints.

## Discussion

*S. agalactiae* infections are more frequent in pregnant women and neonates but are much rarer in non-pregnant adults [1]. However, in some cases, it can present with bacteraemia in non-pregnant adults. Retrospective studies [2,3] and a recent meta-analysis [10] studied some factors predisposing to develop *S. agalactiae* infections and bacteraemia in non-pregnant adults, namely diabetes, malignancies, liver and renal disease and immunosuppressive disorders.

In this case, we report the occurrence of invasive *S. agalactiae* infection in a patient without any known predisposing condition. Furthermore, the involvement of either the central nervous system or joint is exceedingly rare in immunocompetent adults. Large cohort studies and a meta-analysis [5-7] reported *S. agalactiae* as responsible for only 0.4% to 7.4% of all bacterial meningitis. Moreover, the affection of the central nervous system was found to be more frequent in infants and neonates or associated with a predisposing condition such as CSF leakages or extra meningeal sanctuaries, like an abscess or endocarditis. Equally the development of septic arthritis is rare. Large retrospective studies [8,9] showed that *S. agalactiae* is responsible for only 5%-10% of all septic arthritis and is usually linked to a predisposing risk factor as well.

Our patient, despite having no known predisposing risk factor or immunosuppression, developed two unusual manifestations of invasive *S. agalactiae* disease, meningitis, and septic arthritis. To our knowledge, the simultaneous occurrence of these manifestations was only described once in a retrospective study [4].

The occurrence of new symptoms, such as haematochezia and diarrhoea motivated further etiological investigation which enabled us to find the source of this infection, infectious colic ulcers. Both the CNS and articular affection were presumably caused by hematogenous dissemination. Synovial fluid cultures were negative, most likely, due to ongoing directed antimicrobial therapy.

## Conclusions

In conclusion, *S. agalactiae* infection is uncommon in immunocompetent, non-pregnant adults. Furthermore, *S. agalactiae* bacteraemia with CNS or articular involvement is exceedingly rare. A high clinical suspicion, combined with the clinical examination, allows the identification of joint or central nervous system involvement. The early acquisition of blood and fluid cultures allows microbiological identification and prompt treatment initiation, improving the prognosis.
